This article has been retracted.

# Integrated Analysis of miRNA-mRNA Regulatory Networks Associated with Osteonecrosis of the Femoral Head

**DOI:** 10.1155/2021/8076598

**Published:** 2021-08-12

**Authors:** Liwei Yu, Tengfei Yao, Zhoulei Jiang, Tong Xu

**Affiliations:** ^1^Department of Orthopedics, The Second Hospital of Haishu District, Ningbo, China; ^2^Department of Orthopedics, The First Affiliated Hospital of Jiangxi Medical College, Nanchang, China; ^3^Department of Ultrasound, Ningbo Ninth Hospital, Ningbo, China; ^4^Department of Orthopedics, Shangrao Hospital of Traditional Chinese Medicine, Shangrao, China

## Abstract

Osteonecrosis of the femoral head (ONFH) accounts for as many as 18% of total hip arthroplasties. Knowledge of genetic changes and molecular abnormalities could help identify individuals considered to be at a higher risk of developing ONFH. In this study, we sought to identify differentially expressed miRNAs (DEmiRs) and genes (DEGs) associated with ONFH by integrated bioinformatics analyses as well as to construct the miRNA-mRNA regulatory network involving in the pathogenesis of ONFH. We performed differential expression analysis using a gene expression profile GSE123568 and a miRNA expression profile GSE89587 deposited in the Gene Expression Omnibus and identified 47 DEmiRs (24 upregulated miRNAs and 23 downregulated miRNAs) and 529 DEGs (218 upregulated genes and 311 downregulated genes). Gene Ontology enrichment analyses of DEGs suggested that DEGs were significantly enriched in neutrophil activation, cytosol, and ubiquitin-protein transferase activity. Kyoto Encyclopedia of Genes and Genomes pathway enrichment analyses of DEGs revealed that DEGs were significantly enriched in transcriptional misregulation in cancer. DEGs-based miRNA-mRNA regulatory networks were obtained by searching miRNA-mRNA prediction databases, TargetScan, miTarBase, miRMap, miRDB, and miRanda databases. Then, overlapped miRNAs were selected between these putative miRNAs and DEmiRs between ONFH and non-ONFH, and pairs of the DEmiR-DEG regulatory network were finally depicted. There were 12 nodes and 64 interactions for upDEmiR-downDEG regulatory networks and 6 nodes and 16 interactions for downDEmiR-upDEG regulatory networks. Using the STRING database, we established a protein-protein interaction network based on the overlapped DEGs between ONFH and non-ONFH. C5AR1, CDC27, CDC34, KAT2B, CPPED1, TFDP1, and MX2 were identified as the hub genes. The present study characterizes the miRNA profile, gene profile, and miRNA-mRNA regulatory network in ONFH, which may contribute to the interpretation of the pathogenesis of ONFH and the identification of novel biomarkers and therapeutic targets for ONFH.

## 1. Introduction

Osteonecrosis of the femoral head (ONFH), also known as avascular necrosis or aseptic necrosis, is a common but complex disease related to ischemia of the femoral head, which finally destroys the structural integrity of the femoral head [1]. In essence, ONFH refers to death of bone cells caused by the damage of microvascular circulation [2]. Although the occurrence of ONFH in the general population have rarely been reported on epidemiological studies in China, a nationally representative survey estimated that 8.12 million people aged 15 years and over in China were associated with ONFH during 2012-2013 [3]. More evidence have manifested that young adults and middle-aged people, especially male, are prone to suffer from ONFH [4]. Although tons of studies have been performed on the etiology, epidemiology, diagnosis, and treatment of ONFH, the exact origin still remains unclear. Some studies have indicated that the trauma [5] and nontraumatic factors involving corticosteroid use [6], habitual drinking [7], and cigarette smoking [8] were strongly contributed to the prevalence of ONFH.

With the progress of molecular technology, the amount of research studies have observed the genetic factors, such as glutamate receptor gene [9], single nucleotide polymorphisms and transient receptor potential vanilloid 4 gene [10], and nitric oxide synthase 3 gene [11], have been accepted to influence the etiology of ONFH. In recent years, an increasing number of studies have manifested that microRNAs have been directly in the regulation of bone development and regeneration in orthopedic diseases, such as osteosarcoma [12], knee osteoarthritis [13], and lumbar disc herniation [14]. miRNAs are thought to be small noncoding RNAs (18–25 nucleotides), which regulate the stability or translation efficiency of their target mRNAs in a negative way to modulate posttranscriptional gene expression [15]. The crucial roles of miRNAs have been widely confirmed in ONFH. For example, miR-155-5p was found to be significantly downregulated in ONFH samples [16]. miR-148a-3p [17], miR-23b-3p [18], and miR-26a [19] were all reported to play a protective role against ONFH. Recent advancement of genome-wide profiling approaches, such as gene microarray and RNA-sequencing technology, enhances the understanding of miRNA and gene expression profiles in the context of ONFH, providing opportunity to identify novel biomarkers and therapeutic targets for ONFH [20, 21]. However, previous miRNA and gene expression profiles studies in ONFH are limited and focused one or several of the differentially expressed miRNAs (DEmiRs) or differential expressed genes (DEGs); none of them focused on the cooperative miRNA-mRNA regulatory mechanism for the pathogenesis of ONFH. In order to deeply understand the diverse biological processes in bones and figure out the regulation in the pathological mechanism of ONFH, in this study, the differentially expression analysis of miRNA and mRNA in ONFH patients compared to non-ONFH was performed, and explore the construction of potential miRNA-mRNA regulatory networks in ONFH by bioinformatics analysis.

## 2. Materials and Methods

### 2.1. Acquisition of Expression Profiles and Differential Expression Analysis

A gene expression profile GSE123568 and a miRNA expression profile GSE89587 were downloaded from the GEO database. GSE123568 was generated on the GPL15207 platform and included serum samples from 30 steroid-induced osteonecrosis of the femoral head (SONFH) patients and 10 non-SONFH patients. GSE89587 was generated on the GPL21439 platform and encompassed serum samples from 10 trauma-induced osteonecrosis of the femoral head (TIONFH) and 10 healing patients. After background correction, quartile normalization and probe summarization with the limma *R* package, DEGs, and DEmiRs between serum samples of ONFH and non-ONFH patients stood out by analyzing GSE123568 and GSE89587 microarray data with log2 |fold change (FC)| ≥ 1, and an adjusted *p* value less than 0.05 was the cutoff value.

### 2.2. Identification of the DEmiR-DEG Regulatory Network

First, putative miRNA targeting DEGs were obtained from multiple miRNA-mRNA prediction databases including TargetScan (http://www.targetscan.org/vert_71/), miTarBase (http://miRTarBase.cuhk.edu.cn/), miRMap (https://mirmap.ezlab.org/), miRDB (http://mirdb.org/), and miRanda (https://www.cs.kent.ac.uk/people/staff/dat/miranda/). After mapping putative miRNA and DEGs using Cytoscape 3.4.0 software, we obtained pairs of the miRNA-DEG regulatory network. Next, overlapped miRNAs were selected between these putative miRNAs and DEmiRs between ONFH and non-ONFH, and pairs of the DEmiR-DEG regulatory network were finally depicted.

### 2.3. GO Term Enrichment Analysis

GO is an international standard classification system for gene function. GO functional annotation refers to three fields, biological process (BP), cellular component (CC), and molecular function (MF). Each field encompasses various gene items. The biological functions of the DEGs are associated with their enrichments in GO items. Different genes coordinate with each other to perform biological functions, and the most important biochemical metabolic pathway and signal transduction pathway involved in target genes can be determined by significantly enriched GO terms screened with the *p* value ≤0.05 as the cutoff value.

### 2.4. KEGG Pathway Enrichment Analysis

KEGG is an important public database for systematic analysis of gene functions in terms of the networks of genes and molecules. The major component of KEGG is the pathway database that encompasses graphical diagrams of biochemical pathways including most of the known metabolic pathways and some of the known regulatory pathways. KEGG enrichment analysis is performed by the Fisher test based on hypergeometric distribution to calculate the significance level (*p* value) of each pathway. The results of multiple hypothesis tests are corrected and the false positive rate (FDR) is obtained, so as to screen the pathways into which the target genes are significantly enriched. The criterion of significance screening is as follows: *p* value ≤0.05. KEGG was analyzed by the clusterProfiler *R* package.

### 2.5. PPI Network Construction

We mapped the DEGs to the Search Tool for the Retrieval of Interacting Genes (STRING online database, http://string-db.org). Interactions with a medium confidence >0.4 were regarded as significant for hub genes. The integrated regulatory networks were constructed using the Cytoscape plugin cytoHubba.

## 3. Results

### 3.1. Identification of DEGs and DEmiRs between ONFH and Non-ONFH

The volcano plot and heatmap were depicted to visualize DEmiRs between serum samples from 10 ONFH patients and 10 healing patients in the GSE89587 dataset (Figures 1(a) and 1(b)). With log2 |FC| ≥ 1 and an adjusted *p* value less than 0.05 as the cutoff value, a total of 47 DEmiRs consisting of 24 upregulated miRNAs and 23 downregulated miRNAs between ONFH patients and healing patients were identified. After differentially analyzing the GSE123568 dataset with log2 |FC| ≥ 1 and an adjusted *p* value less than 0.05 as the cutoff value, 529 DEGs, 218 upregulated genes, and 311 downregulated genes, between serum samples from 30 SONFH patients and 10 non-SONFH patients were identified (Figures 2(a) and 2(b)).

### 3.2. Functional Enrichment Analyses of DEGs between SONFH and Non-SONFH

To study the functional roles of the DEGs between SONFH and non-SONFH in the GSE123568 dataset, GO enrichment analysis was conducted, and significantly enriched GO terms of DEGs are listed in Figure 3(a). From the enrichment results of the BP category, we found that DEGs were significantly enriched in neutrophil activation (GO: 0042119), neutrophil degranulation (GO: 0043312), vesicle-mediated transport (GO: 0016192), neutrophil activation involved in immune response (GO: 0002283), and neutrophil-mediated immunity (GO: 0002446). For the CC category, DEGs were mainly enriched in cytosol (GO: 0005829), spectrin-associated cytoskeleton (GO: 0014731), secretory granule (GO: 0030141), specific granule (GO: 0042581), and tertiary granule (GO: 0070820). Moreover, in the MF category, DEGs were mostly enriched in ubiquitin-protein transferase activity (GO: 0004842), ubiquitin-like protein transferase activity (GO: 0019787), C–C chemokine binding (GO: 0019957), and superoxide-generating NADPH oxidase activator activity (GO: 0016176).  Figure 3(b) is a circle plot that depicts the top 10 GO terms enriched by the DEGs.

### 3.3. Pathway Enrichment Analyses of DEGs between SONFH and Non-SONFH

Subsequently, KEGG enrichment analysis was performed to study the involvement of the DEGs in most of the known pathways in vivo. It was revealed that the DEGs between SONFH and non-SONFH were significantly enriched in transcriptional misregulation in cancer (hsa05202), viral protein interaction with cytokine and cytokine receptor (hsa04061), malaria (hsa05144), mitophagy-animal (hsa04137), and cell cycle (hsa04110) (Figure 4(a)).  Figure 4(b) is a circle plot that depicts the top 9 KEGG pathways enriched by the DEGs.

### 3.4. Identification of the DEmiR-DEG Regulatory Network

First, we obtained DEGs-based miRNA-mRNA regulatory networks by searching the TargetScan, miTarBase, miRMap, miRDB, and miRanda databases. Then, overlapped miRNAs were selected between these putative miRNAs and DEmiRs between ONFH and non-ONFH and pairs of the DEmiR-DEG regulatory network were finally depicted. There were 12 nodes and 64 interactions for upDEmiR-downDEG regulatory networks (Figure 5(a)) and 6 nodes and 16 interactions for downDEmiR-upDEG regulatory networks (Figure 5(b)). The interaction degrees for the DEmiR-DEG regulatory network represent the number of the interactions between the DEmiRs and DEGs. Those DEmiRs and DEGs with high interaction degrees were identified as hub nodes in the DEmiR-DEG regulatory network. The top 9 DEmiRs and 7 DEGs with high degrees from the DEmiR-DEG regulatory network are given in Tables 1 and 2 .

### 3.5. Construction of the PPI Network

The DEGs were mapped into the STRING database to construct the PPI network. In the PPI network, there were 68 nodes, including 43 downregulated DEGs, 25 upregulated DEGs, and 78 interactions (Figure 6). The hub nodes were C5AR1, CDC27, CDC34, KAT2B, CPPED1, TFDP1, and MX2. C5AR1, CPPED1, and MX2 were upregulated DEGs, and CDC27, CDC34, KAT2B, and TFDP1 were downregulated DEGs between ONFH and non-ONFH.

## 4. Discussion

ONFH is a multifactorial orthopedic disease characterized by decreased blood flow leading to bone cell death [22]. The prevalence of ONFH arises from environmental factors, involving serious trauma, corticosteroid medications, and alcohol intake [2], and genetic elements [10]. However, the original pathogenesis of ONFH remains to be explored. Thus, the investigation of the molecular mechanism involved in ONFH is helpful to develop more effective diagnosis and treatment strategies. In this study, the GSE89587 and GSE123568 datasets were used to indicate regulation of miRNAs and mRNAs in the gene expression of ONFH. In brief, according to the GSE89587 dataset, a total of 47 DEmiRs, consisting of 24 upregulated miRNAs and 23 downregulated miRNAs, were identified in 10 TIONFH and 10 healing patients. In addition, 529 DEGs, involving 218 upregulated genes and 311 downregulated genes, were identified in 30 SONFH patients and 10 non-SONFH patients based on the GSE123568 dataset.

In order to further study the interaction between these DEGs, GO term and KEGG pathways analysis were carried out. The GO functional analysis revealed DEGs were significantly enriched in neutrophil activation, neutrophil degranulation, vesicle-mediated transport, neutrophil activation, and neutrophil-mediated immunity in BP term. As to the CC term, it is observed the DEG was mainly concentrated in the cytoplasm, hemoglobin-related cytoskeleton, secretory granules, specific granules, and third granules. DEGs were mostly in enrichment of ubiquitin-protein transferase activity, ubiquitin-like protein transferase activity, C–C chemokine binding, and superoxide-generating NADPH oxidase activator activity in MF term. The KEGG pathways analysis manifested the DEGs were significantly involved in transcriptional misregulation in cancer, viral protein interaction with cytokine and cytokine receptor, and cell cycle. Previous studies suggested the cell adhesion dysfunction, immune response, inflammatory response, and cytokine receptor interaction were associated with the pathogenesis of intracranial aneurysm [23] and steroid-induced ONFH [24]. MiRNAs is involved in the posttranscriptional regulation of eukaryotic genes and is relevant with the cells of development, metabolism, proliferation, growth, differentiation, and death [25]. In this analysis, the DEGs-based miRNA-mRNA regulatory network was constructed by searching the TargetScan, miTarBase, miRMap, miRDB, and miRanda databases, and it was found 8 upregulated miRNAs, containing hsa-let-7b-5p, hsa-let-7d-5p, hsa-miR-30b-5p, hsa-miR-17-5p, hsa-miR-20a-5p, hsa-miR-92a-3p, hsa-miR-92b-3p, and hsa-miR-584-5p, and hsa-miR-302a-3p as downregulated miRNAs, suggesting miRNA expression profiles in the serum sample, were significantly different between the SONFH and non-SONFH patients. Compared with osteoarthritis patients, the expression of miR-17-5p was decreased in the ONFH group, which was inhibited by the expression of homeobox transcription antisense RNA [26]. It was observed that the expression level of miR-30b-5p in metastatic tumors was significantly higher than that in primary tumors and revealed much higher expression in bone metastases than any other metastases [27]. However, there were limited studies on other miRNAs, such as hsa-let-7b-5p, hsa-let-7d-5p, miR-584-5p, and hsa-miR-302a-3p, in regulation of ONFH, but some other researchers have showed the hsa-let-7b-5p revealed significant upregulation in THP-1 macrophages of patients infected *Mycobacterium tuberculosis* [28], and hsa-let-7d-5p was overexpressed in latent tuberculosis infection [29]. In medulloblastoma patients, reduced miR-584-5p expression was correlated with increased levels of the histone deacetylase inhibitor and eukaryotic translation initiation factor 4E type 3 [30]. In addition, it was explored the hsa-miR-302a-3p downregulation was contributed to potential diagnosis for ischemic stroke [31]. Taken together, it was inferred that hsa-let-7b-5p, hsa-let-7d-5p, hsa-miR-30b-5p, hsa-miR-17-5p, hsa-miR-20a-5p, hsa-miR-92a-3p, hsa-miR-92b-3p, hsa-miR-584-5p, and hsa-miR-302a-3p might be related to the process of ONFH.

According to the PPI network, the hub nodes C5AR1, CDC27, CDC34, KAT2B, CPPED1, TFDP1, and MX2 were identified. It was showed that the C5AR1, CPPED1, and MX2 were upregulated and CDC27, CDC34, KAT2B, and TFDP1 were downregulated in DEGs. The deficiency of C5AR1 was involved in the prevention of colorectal cancer, which suggested that the high expression of C5AR1 might be related to colorectal cancer [32]. The CPPED1 revealed higher expression in caesarean birth than in spontaneous births and was associated with regulation of trophoblasts at full-term delivery [33]. Human MX2 is an important IFN-*α* inducible effector, which was found to restrict the HBV replication [34]. In T lymphoblastic lymphoma study, the CDC27 was revealed overexpressed in T lymphoblastic lymphoma tissues, resulting in poor survival [35]. CDC34 was elevated in tumor tissues and was negatively correlated with prognosis of lung carcinogenesis [36]. It analyzed that the downregulation of TFDP1 was indicated in the endometrium of women with deep infiltrating endometriosis [37]. KAT2B and KAT2A were necessity in growth and differentiation of the cartilage and bone in both zebrafish and mice [38]. The findings we observed indicated that C5AR1, CDC27, CDC34, KAT2B, CPPED1, TFDP1, and MX2 might be potential genes which affected the ONFH pathogenesis.

In conclusion, it was observed that hsa-let-7b-5p, hsa-let-7d-5p, hsa-miR-30b-5p, hsa-miR-17-5p, hsa-miR-20a-5p, hsa-miR-92a-3p, hsa-miR-92b-3p, hsa-miR-584-5p, hsa-miR-302a-3p, cytokine and cytokine receptor interaction, malaria, mitophagy-animal, transcriptional misregulation, and cell cycle might be involved in ONFH procedure, which probably provides a novel strategy of treatment and diagnosis on ONFH. But, some limitations were displayed in this study. Further study was required to identify a deeper correlation in miRNAs and mRNAs expression, and it would be better to investigate relevant downstream molecules in ONFH disease by human tissue specimens and animal models. In addition, further in vitro experiments, such as luciferase reporter gene analysis, need to be further studied.

## Figures and Tables

**Figure 1:** Identification of DEmiRs between ONFH and non-ONFH. (a) The volcano plot showing miRNAs with log2 |FC| ≥ 1 and an adjusted *p* < 0.05 as cutoff values; red dots reflect upregulated DEmiRs (*n* = 24), blue dots reflect downregulated DEmiRs (*n* = 23), and black dots reflect non-DEmiRs. (b) The heatmap showing expression diversity of 47 DEmiRs in the GSE89587; the color from blue to red shows the expression from low to high.

**Figure 2:** Identification of DEGs between ONFH and non-ONFH. (a) The volcano plot showing mRNAs with log2 |FC| ≥ 1 and an adjusted *p* < 0.05 as cutoff values; red dots reflect upregulated DEGs (*n* = 218), blue dots reflect downregulated DEGs (*n* = 311), and black dots reflect non-DEGs. (b) The heatmap showing expression diversity of the top 50 DEGs in the GSE123568; the color from blue to red shows the expression from low to high.

**Figure 3:** GO term enrichment analyses of DEGs between ONFH and non-ONFH. (a) Significant enrichment of DEGs in the BP, CC, and MF categories (the top 15 GO terms for each category are listed). (b) A circle plot that depicts the top 10 GO terms enriched by the DEGs.

**Figure 4:** KEGG pathway enrichment analyses of DEGs between ONFH and non-ONFH. (a) Pathways significantly enriched by the DEGs in the KEGG database; red indicates small *p* value and blue indicates large *p* value; the size of the bubbles indicates the degree of enrichment, and larger bubbles reflect larger gene ratio. (b) A circle plot that depicts the top 9 KEGG pathways enriched by the DEGs.

**Figure 5:** Identification of the DEmiR-DEG regulatory network in ONFH. (a) The upDEmiR-downDEG regulatory network consisting of 12 nodes and 64 interactions. (b) The downDEmiR-upDEG regulatory network including 6 nodes and 16 interactions. The interaction degrees for the DEmiR-DEG regulatory network represent the number of the interactions between the DEmiRs and DEGs.

**Figure 6:** Construction of the PPI network. There were 68 nodes, including 43 downregulated DEGs, 25 upregulated DEGs, and 78 interactions. The lines between two nodes indicate the interaction of two proteins; more lines reflect more key locations in the PPI network. The color indicates the interaction degrees, and deeper color reflects higher degree of interaction.

**Table 1:** The top 9 hub DEmiRs from the DEmiR-DEG regulatory network.

DEmiRs	hsa-let-7b-5p	hsa-let-7d-5p	hsa-miR-30b-5p	hsa-miR-17-5p	hsa-miR-20a-5p	hsa-miR-92a-3p	hsa-miR-92b-3p	hsa-miR-584-5p	hsa-miR-302a-3p
Description	upmiRNA	upmiRNA	upmiRNA	upmiRNA	upmiRNA	upmiRNA	upmiRNA	upmiRNA	downmiRNA
Degree	12	10	8	7	6	6	6	4	4

**Table 2:** The top 7 hub DEGs from the DEmiR-DEG regulatory network.

DEGs	YOD1	PGM2L1	E2F2	NME4	KAT2B	AIDA	RTN1
Description	downmRNA	downmRNA	downmRNA	downmRNA	downmRNA	downmRNA	upmRNA
Degree	8	4	3	3	3	3	3

## Data Availability

The gene expression profile GSE123568 and the miRNA expression profile GSE89587 can be downloaded from the GEO database (https://www.ncbi.nlm.nih.gov/gds/?term=).
